# Application of Intelligent Medical Equipment Management System Based on Internet of Things Technology

**DOI:** 10.1155/2022/9149996

**Published:** 2022-02-23

**Authors:** Wei Ren, Xiaochen Wu

**Affiliations:** ^1^School of Computer and Information Sciences, University of the Cumberlands, Williamsburg, KY 40769, USA; ^2^College of Science and Technology, Bellevue University, Bellevue, NE 68005, USA

## Abstract

The management level of medical equipment is an important index to evaluate the modernization degree of hospitals and it is also the basic element of medical and scientific research work, which plays a key role in the development of medical clinical science. Under the background of the rapid development of modern Internet of Things (IoT) technology, hospitals should be fully aware of the role of Internet of Things technology in hospital medical equipment management. With the increasing demand for refined management of medical equipment in hospitals, the application potential of the Internet of Things technology in medical equipment management has gradually become prominent. The management of medical equipment in a hospital is an important part of the management of the hospital, which is related to the medical level, service quality, and economic benefits of the hospital. In this paper, we have analyzed current problems in the management of medical equipment in hospitals, discussed the application of the Internet of Things technology in the management of medical equipment, and promoted the management of medical equipment to be more intelligent and automated. Experimental results have verified that the proposed scheme could be one of the trustworthy automated systems, preferably technology assisted, for the proper management of the medical equipment particularly in hospitals.

## 1. Introduction

The Internet of Things was first mentioned in the book “the way to the future” written by Bill Gates in 1995, but this new concept was not paid attention to at that time. Until 1999, this concept was put forward again by MIT auto-ID and developed rapidly [1]. It is a network concept, which connects any article with the Internet through information sensing devices, such as radio frequency identification (RFID), infrared sensor, global positioning system, and laser scanner, and exchanges and communicates information to realize intelligent identification, positioning, tracking, monitoring, and management [2]. It is another industrial tide after computer, Internet, and mobile communication network. It is not a subversion of these technological revolutions, but a brand-new technological mode transformation integrates these technological applications and improves the technical requirements [3]. As a quality guarantee for hospital diagnosis and treatment, medical equipment is also a basic condition for teaching, medical treatment, prevention, and scientific research, as a decisive condition and material basic condition for improving the level of medical science and technology [4]. As one of the key sources of various medical information generated by medical institutions, medical equipment, as a guarantee of economic and social benefits, can be realized by medical institutions [5]. With the rapid development of the medical industry, the current medical equipment is more advanced and diversified, and the types and quantities of medical equipment in major hospitals are also increasing [6].

For the management of medical equipment, the traditional manual management has been unable to meet the actual needs. The lack of scientificity in the purchase of equipment, the inability to effectively monitor the use of equipment, and the lack of equipment safety management in the management have a great impact on the improvement of the medical level of the hospital [7]. In order to improve the management level of medical equipment, hospitals need to make full use of modern Internet of Things technology, give play to the value of the Internet of Things technology, and achieve the effect of intelligent equipment management [8]. Medical reform is an important issue in China's current social development. The state has invested a lot of social resources to promote its development and made great progress in medical services, preventive health care, medical system, medical equipment, and many other aspects, in order to better serve the people's livelihood [9]. With the development of modern medical technology, medical equipment has been rapidly popularized. Medical equipment has the characteristics of many kinds, large quantity, long service life, high value, scattered locations, and difficult management. Moreover, the nature of hospitals determines that the use of medical equipment is changing all the time, which puts forward new requirements for the dynamic management of hospitals [10]. Although some hospitals have implemented barcode management, which reduces labor intensity to a certain extent and improves the efficiency of equipment management, there are still problems such as difficulty in equipment positioning and error-prone information, resulting in low work efficiency and high error rate. It is necessary to track and manage the equipment in real time and manage the medical equipment scientifically and effectively [11].

Therefore, the use of advanced information technology means for medical equipment information automatic real-time tracking and positioning is particularly important. On the one hand, it can avoid the omission of equipment inspection and maintenance; on the other hand, it is also conducive to defining the responsibility of medical accidents related to medical equipment, changing the current situation that is difficult to accurately manage medical equipment information, and providing the theoretical basis and practical guidance for hospital monitoring and management [12]. At present, most hospitals' medical equipment management systems are information-based management methods, and information-based management has been greatly optimized and improved based on previous manual management, which has the advantages of simple operation and convenient query. However, with the continuous progress of science and technology, the traditional information-based management systems have gradually become difficult to meet the needs of medical equipment management systems at this stage [13]. On the one hand, the efficiency is not high enough and the function is too simple; on the other hand, it is impossible to control the working state of the equipment in real time [14]. Therefore, it is necessary to use the Internet of Things technology to help users manage equipment in the hospital, improve work efficiency, reduce manual operations, and achieve dynamic management and other purposes [15]. Medical equipment is a “thing”, and the Internet of Things is a self-information expression and management method based on the “thing” itself. Therefore, we can try to use the idea of the Internet of Things to solve several problems in the management of medical equipment [16].

In this paper, we have analyzed current problems in the management of medical equipment in hospitals, discussed the application of the Internet of Things technology in the management of medical equipment, and promoted the management of medical equipment to be more intelligent and automated. Experimental results have verified that the proposed scheme could be one of the trustworthy automated systems, preferably technology assisted, for the proper management of the medical equipment particularly in hospitals. First, it helps to realize the fine management of medical equipment. Second, it helps to reduce management costs and improve management efficiency. Third, it helps to improve the use value of medical equipment resources.

The rest of the paper is formatted as given below.

In the subsequent section, the proposed medical equipment management system, specifically its requirements and implementation plan, is described in detail. In Section 3, Internet of Things technology and medical equipment positioning are described in detail. In Section 4, the Application of Intelligent Medical Equipment Management System which is based on Internet of Things technology is presented in detail. Finally, concluding remarks are given.

## 2. Medical Equipment Management

### 2.1. Requirements of Intelligent Management Platform for Clinical Medical Equipment

Large and medium-sized hospitals or medical institutions have strict requirements for the whole process management of various equipment assets, especially for the management, maintenance, and monitoring of large clinical medical equipment [17, 18]. The management department and user department need to know a lot of equipment information from the beginning of procurement demonstration, including the principle and performance of equipment, suitable scenes, and dimensions. The management system should collect and record this information from the beginning to help managers use it in procurement application, procurement arrangement, installation and commissioning, maintenance, and benefit analysis [19]. The sensory control department and emergency department can understand the equipment operation and maintenance status and the distribution of assets for the first time and quickly and accurately understand the equipment operation and maintenance status, so as to evaluate whether the equipment will cause harm to patients and operators or whether there is a risk of infection. Department staff need to understand the distribution of key rescue equipment, be able to grasp the exact location of the first aid equipment, and analyze and consider the rationality of the layout and the convenience of access [20]. The maintenance status, service quality, asset status, and location information in the equipment management system can help management departments and use departments to promptly propose rectification and optimization suggestions, meet clinical needs, and ensure medical quality and safety [21].

### 2.2. Management Status of Medical Equipment

The management of medical equipment includes the whole process of equipment procurement, delivery, acceptance, storage, registration, use, daily maintenance, and scrapping. This is a complicated process, and various problems will inevitably occur in the management process: equipment positioning, tracking, maintenance, analysis, and inquiry [22]. The user demand of the medical equipment maintenance service recommendation system is to solve the fault problem, and the system needs to finally provide a solution. In addition, the various fault parameters of the system are of a professional nature. Some of these fault parameters are not intuitive, but they can be used from the previous one. The medical equipment failure conditions obtained in the stage are obtained and transformed into corresponding failure conditions.  Table 1 is the attribute list of the maintenance service plan of the simplified version of YDB-III.

Among them, scheme ID represents different fault solutions, represented by P1, P2, and other symbols. There are other attributes such as whether the switch is in good condition and whether the oscilloscope is in good condition. These attributes represent the characteristics of the project, that is, listing all kinds of equipment failures, which is equivalent to describing a type of failure, and associated with the corresponding solution ID to form a knowledge domain.

The knowledge base of medical equipment maintenance service includes fact table and rule table. The fact table includes basic knowledge of medical equipment and expert knowledge related to medical equipment failure. The contents of the fact table are shown in Tables 2 and 3.

Medical equipment does not refer to a separate application entity but also includes various types of computer software required. The medical equipment can be summarized into the following categories: first, the diagnostic equipment category, which includes X-ray diagnostic machinery, ultrasonic diagnostic machinery, endoscopy machinery, and nuclear medicine machinery [23]; second, the category of treatment equipment including nursing machinery, surgical machinery, radiotherapy machinery, nuclear medicine treatment machinery, laser machinery, and dialysis treatment machinery in the ward; finally, auxiliary mechanical equipment, including disinfection and sterilization mechanical equipment, refrigeration mechanical equipment, central suction mechanical equipment, oxygen supply mechanical equipment system, medical data processing mechanical equipment, and medical video photography mechanical equipment [24]. In recent years, with the vigorous development of hospital information construction and the increasing demand of patients for medical services, the number and types of medical equipment have increased significantly, which undoubtedly brings new challenges to medical equipment management personnel [25]. Although many advanced technologies have been widely used in the medical field, intelligent management has not been realized in medical equipment management. This will not only increase the workload of managers, resulting in low management efficiency, but also have management loopholes, which are easy to cause asset loss and other phenomena, which will hinder the construction process of modern hospitals [26].

The procurement of medical equipment is one of the important links in hospital management. A scientific and reliable procurement plan can not only save a large number of medical costs for the hospital but also can better meet the business needs of different departments, thereby improving the hospital's medical service level [27]. However, in the current procurement process of medical equipment, most of the managers of the hospital information department or the responsible people of the corresponding departments make the procurement plan of medical equipment by virtue of their personal experience and then the relevant departments of the hospital audit and unified Bidding Procurement [28]. In this case, because it is impossible to dynamically analyze the data of medical equipment in real time, such as the information of the loss degree of existing medical equipment, it is easy to repeatedly purchase or purchase medical equipment, which cannot meet the actual business needs, resulting in waste of medical resources and increasing the operating costs of hospitals [29]. The long-term high-frequency operation can easily cause medical equipment to malfunction or accelerate the rate of aging. Therefore, real-time quality monitoring of medical equipment is necessary. However, the current traditional manual management model is difficult to obtain the operation data of all medical equipment in time. In this case, even if the hospital regularly arranges professional and technical personnel to maintain and repair the medical equipment, it is easy to have safety hazards, which will affect the hospital. The quality of service is shown in [30].

## 3. Internet of Things Technology and Medical Equipment Positioning

### 3.1. Internet of Things Technology

The Internet of Things is an important part of the new generation of information technology. It is a kind of network that connects any article with the article and the article with the network through information sensing devices such as radio frequency identification, infrared induction, global positioning system, and laser scanning, for information exchange and communication, and realizes intelligent identification, positioning, tracking, monitoring, and management of articles. The classification of IoT technology structure is shown in Figure 1.

The Internet of Things technology provides new ideas for the intelligent management of medical equipment. It realizes the information interaction and seamless connection between people and things, and things and things, and achieves the purpose of real-time monitoring, precise management, and equipment sharing of medical equipment. Because the Internet of Things is based on the idea of the Internet and integrates the technologies of various industries, in response to this, the idea of the Internet of Things to solve problems in the industry is also a hot spot in today's technological development. In the application of various industries, the Internet of Things has three advantages: concept advantage, technical advantages, and policy advantages. Compared with radio frequency identification technology, the intelligent sensor does not need to set a specific tag, which can control the cost to a large extent, but this technology also has some defects. When using intelligent sensing technology to obtain the corresponding characteristics of data information, the key is the inductive chemical, physical, and biological characteristics. At present, infrared technology is widely used, resulting in its function being greatly limited. Based on this technology, this technology has realized various recognition modes, such as face recognition technology and fingerprint recognition technology, and promoted many changes in national life and production.

### 3.2. Medical Equipment Positioning System Hardware

The equipment location and secondment business mean that users can check the location of the access device through the system and make secondments according to their needs. Take equipment positioning and secondment as an example. The business process is shown in Figure 2. After the user logs in to the system, he can obtain the device location by viewing the positioning function. At this time, the user can second the equipment according to the actual situation. After submitting the secondment application, he can contact the asset The administrator conducts secondment-related work with the equipment administrator of the system.

The indoor positioning system of medical equipment needs the cooperation of positioning hardware system, positioning data server, and user mobile terminal application App. According to the requirements of the front analysis of medical equipment indoor positioning and tracking requirements, designed for positioning hardware module, positioning server module, and user terminal application module, the user terminal application module is composed of code scanning registration, medical equipment positioning information, and indoor working environment.

Among them, the indoor positioning system is composed of positioning reference ZigBee node, WiFi base station, and mobile tag node of medical equipment. These systems are responsible for collecting RSSI (received signal strength indication) values of ZigBee reference nodes and mobile tag nodes and forwarding them to the positioning data server. The user's mobile terminal uses App to scan the QR code attached to the mobile medical equipment and binds it to the mobile positioning tag nodes. The mobile terminal App is used to locate the fixed medical equipment through the indoor wireless network to obtain the RSSI data of the positioning target medical equipment and the current positioning reference ZigBee node from the server, and the server service program runs the positioning algorithm to calculate the accurate position of the medical equipment. When the mobile medical device is located, the mobile node sends a signal to the reference node, and the reference node receives the signal to feed back the mean value of RSSI in the period to the location coordinator. The location coordinator of the mobile node receiving the feedback signal sends the RSSI value to the location server to calculate the location result.

The cooperation flow of the positioning hardware system, the positioning data server, and the user mobile terminal application App is shown in Figure 3.

The node size of the positioning hardware system is determined according to actual needs. The basic requirements are as follows: several ZigBee nodes are used as positioning reference nodes, and a ZigBee node is attached to medical equipment as a mobile tag node. The positioning server obtains the positioning data from the positioning coordinator through WiFi wireless interface, decomposes the data sequence composed of RSSI values, and writes the results into the positioning database. The database data analysis and processing function are realized based on ASP. NET and finally can be displayed graphically.

The above hardware collects effective data for the positioning of medical devices. The positioned device exchanges data with the nearest receiver through the RFID chip. The receiver position is uniformly coded. The collected data is calculated on the server-side through the trilateral positioning algorithm to obtain the building and floor and location information of the equipment to be located and display the specific location on the user terminal to realize the positioning function of the medical equipment.

Trilateration is a common location algorithm: it is known as three points shown in Figure 4, known three-point position (*x*_1_, *y*_1_), (*x*_2_, *y*_2_), (*x*_3_, *y*_3_) takes *d*_1_, *d*_2_, *d*_3_ as radius as three circles, and according to Pythagoras theorem, the calculation formula of the intersection point is unknown point position:


(1) $$\begin{array}{c} {\left(x_{1}-x_{0}\right)}^{2}+{\left(y_{1}-y_{0}\right)}^{2}=d_{1}^{2},\\ {\left(x_{2}-x_{0}\right)}^{2}+{\left(y_{2}-y_{0}\right)}^{2}=d_{2}^{2},\\ {\left(x_{3}-x_{0}\right)}^{2}+{\left(y_{3}-y_{0}\right)}^{2}=d_{3}^{2}. \end{array}$$

The three-side positioning principle diagram is shown in Figure 5.

Let the unknown point be (*x*, *y*), so that the coordinates of the first spherical *P*_1_ are (0, 0), *P*_2_ is in the same ordinate, the coordinates of the spherical center are (*d*, 0), *P*_3_ is (*I*, *j*), the radii of the three spheres are *r*_1_, *r*_2_, *r*_3_, and *z* is the height between the intersection point of the three spheres and the horizontal plane. There are

(2) $$\begin{array}{c} r_{1}^{2}=x_{2}+y_{2}+z_{2},\\ r_{2}^{2}={\left(x-d\right)}^{2}+y^{2}+z^{2},\\ r_{3}^{2}={\left(x-i\right)}^{2}+{\left(y-j\right)}^{2}+z^{2}. \end{array}$$

When *z* = 0, it means that the three circles intersect at a point on the horizontal plane. First, solve for *x*:

(3) $$\begin{array}{c} x=\frac{\left(r_{1}^{2}-r_{2}^{2}+d^{2}\right)}{2\;d},\\ y=\frac{\left(r_{1}^{2}-r_{3}^{2}-x^{2}+{\left(x-i\right)}^{2}+j^{2}\right)}{2j}. \end{array}$$

The coordinates of a relatively accurate point (*U*) can be obtained through calculation, and the coordinates of the moving target can be calculated. Then, the positioning interface of the medical device realizes map management based on the underlying image processing technology and uses the weighted centroid positioning algorithm and the optimized weighted centroid positioning algorithm to pair. The positioning of the target node can once again improve the positioning accuracy. The classes required by the user terminal application include the entity classes used to represent the positioning of medical equipment. The requirements are shown in Table 4.

Table 5 shows the action requirements of the medical device positioning response applied by the user terminal.

According to the specific application environment of medical equipment, the positioning database is designed as an optimal database mode, so as to meet the diversified application requirements of various users. There are five fields in the medical table. They are id (number), name (equipment name), function (equipment function), environment (equipment working environment), and image (equipment sample drawing), as shown in Table 6.

## 4. Application of Intelligent Medical Equipment Management System Based on Internet of Things Technology

### 4.1. The Application of Internet in Medical Equipment Management

The intelligent management system structure of medical equipment based on the Internet of Things includes three layers: perception layer, network layer, and application layer. The bottom layer is the perception layer, which mainly perceives objects through automatic identification technologies, such as RFID and sensors, and collects dynamic and static data information such as device identity information and environmental status. The middle layer is the network layer for data transmission. It mainly transmits the sensed information safely and reliably through the network to achieve interconnection. The top layer is the application layer, which is the interface between the Internet of Things and users. Only by combining it with the needs of each industry can the intelligent application of the Internet of Things be realized. In the intelligent management system of the hospital, the LAN of the hospital is used as the main body of the network transmission layer, which connects all kinds of devices in the perception layer downward and the medical equipment management platform upward to realize the intelligent management of information. The architecture of the system is shown in Figure 6.

The core of the Internet of Things is the Internet of Things. Equipment management based on the Internet of Things transforms the traditional manual management of equipment into self-management of equipment, which is more efficient and reliable in terms of management effect. Its advantages are mainly reflected in the following aspects. Equipment records are efficient and have high quality. Scientific evaluation of equipment usage, reuse equipment to save resources, telemonitoring medical equipment, and home care medical equipment are shown in Figure 7 in the use of the Internet of Things technology in smart medical care, under normal circumstances, and monitor the physiological parameters of the monitored object. If an accident occurs, it needs to be rescued in time. The physiological data of the human body can be collected into the sensor device and transplanted into the life sensor of the human body so that the two can form a whole wireless network together, which is the key component and sensing part of the Internet of Things.

Most of the nosocomial infections were caused by poor disinfection. As one of the key departments to control nosocomial infection, disinfection and supply room play a vital role. In the intelligent disinfection supply tracking system, the whole process of the disinfection package is traced based on the wireless network, wireless mobile terminal equipment, and a two-digit bar code. At the same time, record the disinfection process monitoring of operators, as shown in Figure 8.

### 4.2. Algorithm Research of Voice Command Control System Suitable for Medical Equipment

According to industry forecasts, in healthcare services, the demand for various diagnostic services will grow rapidly in the next ten years. Due to the shortage of manpower, the urgent requirements for quick and economical inspections, and the lack of qualified operators, putting more and more pressure on clinical diagnosis, clinicians have always hoped to achieve a revolutionary leap in instrument performance and workflow.

The speech recognition system is essentially a pattern recognition system, and its basic structure is shown in Figure 9. The speech signal is collected by a computer and the characteristic parameters of speech are analyzed. Then, these features are stored in the computer and used as the speech test template in the speech parameter library. This process is called “training”. Next, the voice to be recognized is collected by the computer, and the voice feature parameters to be recognized are obtained through the same analysis process as that during training. Then, it is compared with the reference templates in the library one by one, and the template closest to the voice feature to be recognized is found by a certain judgment method. When the recognition result is obtained, this process is called “recognition”. The standard for comparison is to measure the “distortion measure” between speech parameter vectors.

The digitization of the voice signal is to transform the analog signal into a digital signal with discrete time and amplitude, including sampling and quantization.

#### 4.2.1. Sampling

Sampling is to discretize the time-continuous signal *s*(*t*) into a sample sequence *s*(*n*) = *s*(*nT*), *T* is the sampling period, and its reciprocal is called the sampling frame rate.

The following parameters are optional:

1. Sampling frequency: 8.000 khz,11.025 kHz, 12.000 kHz, etc.
2. Sampling accuracy: 8 bits, 16 bits, etc.
3. Number of channels: mono, two-channel stereo, etc. The sampled file is saved in. wav format.

#### 4.2.2. Quantization

We discretize the sample amplitude in the sample sequence. That is, one of a limited number of values approximately represents the sampled value of the waveform. If the signal range is |*s*(*n*)| ≤ *S*max, in order to effectively use the binary code, the peak-to-peak range is generally expressed as

(4) $$\begin{array}{c} 2S\max=\Delta 2^{B}. \end{array}$$

In the formula, Δ stands for quantization, and 2^*B*^ stands for a level number. The error *c*(*n*) between the quantized value and the original analog value is called quantization noise. According to Δ and B, the quantization noise can be expressed as

(5) $$\begin{array}{c} -\frac{\Delta }{2}\leq c\left(n\right)\leq \frac{\Delta }{2}. \end{array}$$

Determination of sampling parameters.

  Sampling: the microphone is connected to the computer sound card for sampling.
  Sampling rate: 11.025 kHz
  Sampling accuracy: 16 bits, etc.
  Number of channels: mono.
  The sampled file is saved in. wav format.

Next, the windowing and framing processing will be carried out. Generally, the number of frames per second is about 33∼100 frames, depending on the actual situation. Although the method of continuous segmentation can be adopted for framing, the method of overlapping segmentation as shown in Figure 10 is generally adopted, in order to make the transition between frames smooth and maintain its continuity. The overlapping part of the previous frame and the next frame is called frameshift. The ratio of frameshift to frame length is generally 0∼1/2. Framing is achieved by weighting with a movable window of finite length, which is to use a certain window function *w*(*n*) to multiply *s*(*n*) to form a windowed speech signal *s*_*w*_(*n*)=*s*(*n*) × *w*(*n*). There are two commonly used window functions.

Rectangular window:

(6) $$\begin{array}{c} w\left(n\right)\left\{\begin{array}{cc} 1, & \left(0\leq n\leq N-1\right),\\ 0, & \left(n=\text{else}\right). \end{array}\right) \end{array}$$

Hamming window:

(7) $$\begin{array}{c} w\left(n\right)\left\{\begin{array}{cc} 0.54-0.46\;\cos\left[2\pi \frac{n}{N-1}\right], & \left(0\leq n\leq N-1\right),\\ 0, & \left(n=\text{else}\right). \end{array}\right) \end{array}$$

The following relationships exist between the length of the sampling period *T*_*s*_=1/*f*_*s*_, the window length N, and the resolution Δ*f* of the window:

(8) $$\begin{array}{c} \Delta f=\frac{1}{{\text{NT}}_{s}}. \end{array}$$

Although different short-term analysis methods (time-domain analysis, frequency domain analysis, and inverse domain analysis) and different speech feature parameters may have different requirements for window function, generally speaking, the standard of a good window function is as follows: in the time domain, because it is the speech waveform multiplied by the window function, it is necessary to reduce the slope at both ends of the time window and make the two ends of the window edge smoothly transition to zero without causing sharp changes, so that the intercepted speech waveform can be slowly reduced to zero and the truncation effect of speech frames can be reduced. In the frequency domain, it is necessary to have a wide bandwidth and a small maximum sideband. Here, only the typical rectangular window and Hamming window are compared.

(9) $$\begin{array}{c} \text{Rectangular window }h\left(n\right)\left\{\begin{array}{cc} 1, & 0\leq n\leq \left(N-1\right),\\ 0, & n=\text{else}. \end{array}\right) \end{array}$$

The frequency response of the digital filter corresponding to the unit function response is

(10) $$\begin{array}{c} H\left(e^{\text{JWT}}\right)=\sum_{n=0}^{N-1}e^{-\text{JWT}}\\ =\frac{\sin\left(\text{NWT}/2\right)}{\sin\left(\text{WT}/2\right)}e^{-\text{JWT}\left(N-1\right)/2}. \end{array}$$

It has a linear phase-frequency characteristic and the corresponding frequency when its frequency characteristic is the first zero value.

(11) $$\begin{array}{c} f_{01}=\frac{f_{s}}{N}\\ =\frac{1}{{\text{NT}}_{s}}. \end{array}$$

Here, *f*_*s*_ is the sampling frequency and *T*_*s*_=1/*f*_*s*_ is the sampling period.

(12) $$\begin{array}{c} \text{Hamming window }h\left(n\right)\left\{\begin{array}{cc} 0.54-0.46\;\cos\left[2\pi n/\left(N-1\right)\right], & \left(0\leq n\leq N-1\right),\\ 0, & n=\text{else}. \end{array}\right) \end{array}$$

It is found that the first zero frequency (bandwidth) of the frequency response *H*(*e*^JWT^) and the attenuation outside the passband are much larger than those of the rectangular window. Some reference data of rectangular window and Hamming window are shown in Table 7.

From Table 1, we can see that the main discrimination width of Hamming window is twice as large as that of the rectangular window, that is, the bandwidth is doubled, and its out-of-band attenuation is more than twice as large as that of the rectangular window. The spectral smoothing performance of a rectangular window is better, but the high-frequency components are lost, which makes the waveform details lost. The Hamming window is the opposite. From this point of view, the Hamming window is more suitable than the rectangular window. At the same time, considering that the latter algorithm needs to use FFT because it cannot guarantee that the signal cut out is exactly one cycle, if the time window of the attenuation type at both ends is not used, the signals (discontinuities) at both ends will affect the spectral characteristics, resulting in the fact that the spectrum is unstable. Therefore, in order to weaken this effect, a window function of attenuation at both ends is required.

## 5. Conclusion

The application of the intelligent medical Internet of Things can realize the interconnection between people and things. The data of different dimensions of multiple objects are gathered into a large amount of data. The Internet of Things technology is used to further mine these data and comprehensively detect and analyze various health risk factors. Through the remote wireless health management service platform, the difficulty of seeing a doctor can be greatly alleviated. Intelligent management of medical equipment based on the Internet of Things has truly realized the digitalization and mobility of hospital information. In the design of instruction content, we should not only examine the humanization of instruction but also consider whether instruction design can reduce the trouble for the system identification process. The continuous development of medical equipment and the major changes in equipment brand types, clinical functions, and structural performance have put forward new requirements for the equipment management capabilities of medical engineering and technical personnel. Establishing job competency standards for medical engineering and technical personnel, building a cooperation platform between the government, industry, and hospitals, standardizing professional behaviors, and improving management standards can provide institutional guarantees for the modern management of hospitals.

## Figures and Tables

**Figure 1:** Classification of the IoT technology structure.

**Figure 2:** Flow chart of equipment positioning and secondment business.

**Figure 3:** Positioning workflow.

**Figure 4:** Three-side positioning principle diagram.

**Figure 5:** Three-side positioning principle diagram.

**Figure 6:** Architecture diagram.

**Figure 7:** Application of IoT technology in smart healthcare.

**Figure 8:** Sterilization supply room tracking system.

**Figure 9:** The composition of the speech recognition algorithm system.

**Figure 10:** Windowing and framing of the speech signal.

**Table 1:** Maintenance service plan of simplified version equipment.

Plan id	Display screen	Power supply fan	CZ5 Pin 4	CZ5 Pins 1, 3	CZ5 Resistance	8031/8155 Pins
P1	1	2	2	1	1	2
P2	1	2	1	1	1	1

**Table 2:** Fact table parameter description.

Field name	Type of data	Description
Display screen	boo1	Whether the display shows
Power supply fan spinning	boo1	Whether the power supply fan rotates
CZ5 pin 4	boo1	Whether the pin has 5 V
CZ5 pins 1, 3	boo1	Whether the pin has +12 V
CZ5 resistance	boo1	Whether short circuit, refer to 70 ohm
8031/8155 pins	boo1	Whether the pin has 5V

**Table 3:** Fact table design.

Plan id	Display screen	Power supply fan	CZ5 Pin 4	CZ5 Pins 1, 3	CZ5 Resistance	8031/8155 Pins
P1	1	2	2	1	1	1
P2	1	2	1	1	1	1

**Table 4:** Medical equipment positioning category.

Class name	Class file	Attributes
Round	Circle.java	*X* coordinate, *y* coordinate, radius
Medical equipment	Cutral.java	Number, name, picture address collection, function introduction
Reference point information	ReferencePoint. java	*X* coordinate, *y* coordinate
Positioning analysis conclusion	Result.java	Number of results, coordinate point
Reference node	Sensor. java	Reference node number, area number, positioning data

**Table 5:** Positioning response actions.

Action name	Class name	Effect
Medical device registration	Register. java	Scan the QR code and register the medical device
Mobile label node location information	ReferenceInfo.java	Show the time change of the sensor's data
Medical equipment positioning	MedicalEquipment. java	Give medical equipment positioning information
Location response	LocFeedback. java	Give feedback on medical device positioning
Reference node assisted positioning	SensorsAuxiliary.java	Reference node information required for positioning

**Table 6:** Medical table.

Field name	Category	Primary key	Nonempty
ID	Int	Yes	Yes
Name	Varchar (5o)	No	Yes
Function	Varchar (500)	No	Yes
Environment	Varchar (5o0)	No	Yes
Descriptions	Image	No	Yes

**Table 7:** Comparison of the rectangular window and Hamming window.

Window type	Sidelobe peak	Peak value	Minimum stopband attenuation
Rectangular window	−24	4*π*/*N*	−32
Hamming window	−52	8*π*/*N*	−64

## Data Availability

The data used to support the findings of this study are included within the article.

## References

[1] Ni L., Xue P., An C. (2021). Establishment of normal range for thromboelastography in healthy middle-aged and elderly people of weihai in China. *Journal of Healthcare Engineering*.

[2] Xiao L., Liao J., Hong Y., Yan Z. (2020). Research on the design and application of intelligent rental system for medical equipment in use in hospitals based on Internet of things technology. *China Medical Equipment*.

[3] You C., Gong Q., Huang Y., Weihua P. (2020). Construction and practice of a hospital-level medical equipment data collection management platform based on Internet of Things technology. *China Medical Equipment*.

[4] Gong H. (2020). Research on the application of Internet of things technology in medical equipment management. *Information and Computer (Theoretical Edition)*.

[5] Song J., Mou Q., Guo H. (2020). Research and application of large-scale medical equipment safety monitoring system based on Internet of Things technology. *Medical Equipment*.

[6] Wang X. (2016). Design of handheld medical equipment archives management system based on Internet of things. *Archives and Construction*.

[7] Gao F., Zhang S., Liu H. (2016). Design of medical equipment condition monitoring system based on Internet of Things technology. *China Medical Equipment*.

[8] Fang Z. (2020). The design of an intelligent well management system based on the Internet of Things. *China Cable TV*.

[9] Cao H., You J., Zheng Y., Chen Y., Li B., Chen M. (2018). Practice and exploration of a regional medical equipment cloud management platform based on the Internet of Things. *Chinese Journal of Medical Devices*.

[10] Wang Z., Guo H., Gan M., Chang F., Li B. (2020). Analysis of progress in medical equipment information management. *Biomedical Engineering and Clinics*.

[11] Pan Z. (2019). Research on the management of large-scale medical equipment in the construction of smart hospitals. *Food & Health*.

[12] Chen J., Wei H., Qin L., Zhou J. (2020). Application of Internet of Things technology in lean cost management of medical equipment in operating room. *China Medical Equipment*.

[13] Qiu D. (2017). Discussion on the application of Internet of Things technology in medical equipment management. *Smart Health*.

[14] Wan Li, Wang D., Guo J. (2018). Research on online monitoring and life cycle prediction of medical equipment based on Internet of Things technology. *Modern Hospital Management*.

[15] Zhang H. (2019). The application of IoT technology in the management of medical equipment in the 5G era. *China New Telecommunications*.

[16] Liu H., Ma L. (2017). Exploration of medical equipment management based on Internet of Things technology. *Science & Technology Communication*.

[17] Chu M. (2018). The application of Internet of Things technology in medical equipment. *Digital Technology and Application*.

[18] Pan J (2016). Intelligent management platform for medical equipment management and fault maintenance. *Medical Equipment*.

[19] Xiang P., Liu Y., Chen L., Liu Y. (2018). Development and application of medical equipment and consumables management system interacting with hospital computer business system. *China Medical Equipment*.

[20] Shen Y., Shen Z., Dang H. (2021). Design and implementation of a shared management system for medical equipment. *China Medical Equipment*.

[21] Wang Z., Jin Z. (2020). Architecture and function design of medical equipment management system. *Information Recording Materials*.

[22] Yahu W. (2018). Construction of medical equipment measurement quality control information management system. *Great Doctor*.

[23] Liao M., Zhen W., He C. (2018). Fine management of medical equipment based on the integration of resource allocation. *Medical Equipment*.

[24] Du Z., Wang M., Liu S., Fan J., Zu H. (2017). Design and application of smart medical equipment cabinet based on RFID technology. *China Medical Equipment*.

[25] Shi L. (2016). Maintenance and repair of computer software systems in medical equipment. *Digest of World Latest Medical Information*.

[26] Wang W., Zhang H., Quan H. (2016). Discussion on the intelligent development trend and safety control strategy of medical equipment. *Medical and Health Equipment*.

[27] Zhang C. (2018). Management and maintenance technology of computer components in medical equipment. *Science and Technology Wind*.

[28] Du H. (2018). Talking about the management of medical equipment in our hospital. *Digest of World Latest Medical Information*.

[29] Pu Y. (2020). Discussion on a new equipment management framework based on the Internet of Things technology. *Modern Business and Trade Industry*.

[30] Gao F., Zhang S., Liu H., Yang Y., Ma C., Tang Y. (2016). Design of precise positioning system for medical equipment based on Internet of Things technology. *China Medical Equipment*.

